# Risk Factors for Dupuytren's Contracture: A Case-Control Study

**DOI:** 10.1155/2022/3574037

**Published:** 2022-04-28

**Authors:** Liangxiao Zheng, Dongliang Chen, Peng Liu, Jinwei Liu, Xiaofeng Song, Zengfang Zhang

**Affiliations:** Department of Hand and Foot Surgery, Qilu Hospital (Qingdao), Cheeloo College of Medicine, Shandong University, 758 Hefei Road, Qingdao, Shandong 266035, China

## Abstract

**Objective:**

To study the risk factors of Dupuytren's contracture (DC) and to provide a reference for the clinical prevention and treatment of DC.

**Methods:**

The clinical data of 21 DC patients treated with surgery in Qilu Hospital of Shandong University (Qingdao) from March 2014 to January 2022 were collected. During the same period, 31 subjects who were admitted to the hospital for treatment of finger numbness, difficulty in movement, and other reasons were selected as the control group, and the clinical data of the control group were collected. A case-control study was used to analyze the risk factors for DC. The receiver operating curve (ROC) was used to analyze the efficacy of blood biochemical indexes and coagulation-related indexes in predicting the occurrence of DC.

**Results:**

Multivariate logistic regression analysis showed that male and diabetes were independent risk factors for the occurrence of DC (HR = 19.69, 95%CI: 3.12–124.19, *P* = 0.002; HR = 7.61, 95%CI: 1.25–46.47, *P* = 0.03). The results of the ROC analysis showed that the area under the curve (AUC) for the DC predicted by cystatin C was 0.7565 (95%CI: 0.6203–0.8928, *P* = 0.0018), and the AUC for the DC predicted by blood chloride level was 0.8121 (95%CI: 0.6880–0.9362, *P* = 0.0002), the AUC for the DC predicted by fibrinogen was 0.7796 (95%CI: 0.6439–0.9152, *P* = 0.0007), the AUC for the DC predicted by D-dimer level was 0.8740 (95%CI: 0.7812–0.9669, *P* < 0.0001), and the AUC for the DC predicted by thrombin time was 0.7803 (95%CI: 0.6411–0.9196, *P* = 0.0007). The AUC for the DC predicted by the combined detection of cystatin C, blood chloride, fibrinogen, D-dimer, and thrombin time was 0.9441 (95%CI: 0.8926–0.9957, *P* < 0.001).

**Conclusion:**

Male and diabetes are independent risk factors for the occurrence of DC. Combined detection of cystatin C, blood chloride, fibrinogen, D-dimer, and thrombin time has a certain value in predicting the occurrence of DC.

## 1. Introduction

Dupuytren's aponeurosis is located in the middle of the palm and is a triangular fascia-like tissue under the skin, covering the surface of the flexor digitorum tendon and the earthworm-like muscle [1]. Since the 18th century, many researchers have carried out a lot of research on Dupuytren's disease (DC), but there is still no clear conclusion on the pathogenesis of DC, and its treatment is mainly surgery [2, 3]. In recent years, with the improvement of Chinese people's living conditions and medical standards, the popularization of medical and health care knowledge, and the improvement of patients' requirements for aesthetics, the demand for DC diagnosis and treatment in China is also increasing.

Although the etiology of DC is still unclear, many etiologies related to cellular and connective tissue changes have been identified, which may be related to ethnic factors, trauma factors, genetic factors, and environmental factors. For example, DC is more common in European and American countries, but less common in Asian countries [4]. In a retrospective study of approximately 10,000 U.S. veterans, the incidence was approximately 734/100,000 for whites, 1.30/100,000 for blacks, 237/100,000 for white Hispanics, and 144/100,000 for native Americans, the incidence rate of the yellow race was only 67/100,000 [5]. Some researchers retrospectively analyzed the data of 385 patients with DC secondary to trauma or surgery and found that patients can suffer from the disease within 1 year after injury, and the earliest nodules or cords appear in the injured palm [6]. Therefore, trauma is also considered to be one of the contributing factors to the morbidity of susceptible people. Some researchers studied the clinical data of 92 DC patients and found that patients with younger ages and patients with severe symptoms were mostly accompanied by a clear family history, and the influence of genetic factors was stronger than that of environmental factors [7].

At present, surgery is still the main treatment option for DC. In the case of surgical pointers, early surgery is easy to correct the deformity. Although several risk factors for the occurrence of DC have been reported by researchers, including smoking, hypertension, genetic factors, and diabetes [8–11], the specific pathogenesis and exact etiology are still controversial. Recently, the incidence of DC has received less attention from researchers due to its low incidence in the Chinese population.

Therefore, we focused on analyzing the clinical data of DC patients and compared it with the clinical data of non-DC control subjects to analyze the risk factors for the occurrence of DC in this study.

## 2. Materials and Methods

### 2.1. Subjects

A total of twenty-one DC patients treated with surgery in Qilu Hospital of Shandong University from March 2014 to January 2022 were selected for this study. Inclusion criteria: (1) patients with a definite diagnosis of palmar DC; (2) nodules, cords, and finger contracture deformities characteristic of palmar DC; and (3) surgery has been performed. Exclusion criteria: (1) patients with general scar contracture of the hand and congenital polyarticular contracture; (2) patients with flexion deformity of the fingers caused by Dupuytren's contracture and scar contracture that cannot be differentiated; and (3) patients without surgical treatment. This study was approved by the Ethics Committee of Qilu Hospital of Shandong University (Qingdao) (KYLL-2022004), and all subjects signed informed consent.

### 2.2. Clinical Data

In this study, we collected the subjects' basic clinical data, including age, gender, height, weight, body mass index (BMI), smoking history, drinking history, hypertension history, diabetes history, and coronary heart disease history. According to the blood biochemical results of the subjects admitted to the hospital, we collected the subjects' albumin, cystatin C, creatinine, alanine aminotransferase, aspartate aminotransferase, total bilirubin, direct bilirubin, indirect bilirubin, total bile acids, total cholesterol, triglycerides, high-density lipoprotein cholesterol (HDL-C), low-density lipoprotein cholesterol (LDL-C), glucose, blood urea nitrogen, creatinine, uric acid, potassium, sodium, and chlorine. And the detection results of coagulation-related indicators such as fibrinogen, D-dimer, and thrombin time were also collected.

### 2.3. Statistical Analysis

In this study, IBM SPSS Statistics (version 26, R26.0.0.2, IBM, Chicago, USA) and GraphPad Prism (version 8.4.0, GraphPad Software, USA) were used for statistical analysis in this study. Continuous variables with normal distribution were shown as mean ± standard deviation, and differences were analyzed by *t*-test or one-way ANOVA. Categorical variables were shown as frequencies (*n* (%)), and differences between the two groups were analyzed using the *χ*^2^ test. Logistic regression was used to analyze the risk factors for the occurrence of DC, and the influence of other confounding factors was adjusted. The receiver operating curve (ROC) was used to analyze the efficacy of blood biochemical parameters and coagulation-related parameters in predicting DC, and the area under the curve (AUC) was calculated. An estimated 22 cases in the DC group and 32 cases in the control would be needed to provide 80% power for multivariate logistic regression analysis results. All assays were two-tailed, and *P* < 0.05 indicated a statistically significant difference.

## 3. Results

### 3.1. Clinical Information

The clinical data of DC patients and control subjects are shown in Table 1. The results of the univariate analysis showed that among the included subjects, the proportions of male patients, smokers, and diabetes patients in DC patients were significantly higher than those in the control group, and the differences were statistically significant (*P* < 0.05). There was no significant difference in the proportion of patients with coronary heart disease between DC patients and the control group (*P* > 0.05).

### 3.2. Analysis of Risk Factors for the Occurrence of DC

Multivariate Logistic regression was used to analyze the risk factors for the occurrence of DC, and the results are shown in Table 2. We found that male gender and diabetes were independent risk factors for the occurrence of DC (HR = 19.69, 95%CI: 3.12–124.19, *P* = 0.002; HR = 7.61, 95%CI: 1.25–46.47, *P* = 0.03).

### 3.3. Correlation between Blood Biochemical Levels and DC

The blood biochemical index levels of DC patients and control subjects were analyzed and compared, the results are shown in Table 3. We found that the level of cystatin C in the blood of DC patients was significantly higher than that of the control group, and the chloride ion level was significantly lower than that of the control group, and the differences were statistically significant (*P* = 0.032, *P* < 0.001).

### 3.4. ROC of Blood Biochemical Indexes to Predict DC

We analyzed the receiver operating curve (ROC) of blood biochemical indicators for predicting DC, and calculated the area under the curve (AUC), the results showed that the AUC of cystatin C for predicting DC was 0.7565 (95%CI: 0.6203–0.8928), *P* = 0.0018. The AUC of blood chloride level for predicting DC was 0.8121 (95%CI: 0.6880–0.9362) (*P* = 0.0002) (Figure 1).

### 3.5. The Relationship between Blood Coagulation-Related Indexes and DC

The levels of coagulation-related indexes in DC patients and control subjects were analyzed and compared, and the results are shown in Table 4. The coagulation-related indicators we analyzed included fibrinogen, D-dimer, and thrombin time. The results showed that the levels of fibrinogen and D-dimer in DC patients were significantly lower than those in the control group, and the thrombin time was significantly longer than that in the control group, the differences were statistically significant (*P* < 0.01).

### 3.6. ROC of Coagulation-Related Indicators for Predicting DC

We analyzed the receiver operating curve (AUC) of different coagulation-related indicators in DC patients and controls for predicting DC. The analysis results showed that the AUC of fibrinogen for predicting DC was 0.7796 (95%CI: 0.6439–0.9152), *P* = 0.0007. The AUC of D-dimer level predicting DC was 0.8740 (95%CI: 0.7812–0.9669), *P* < 0.0001. The AUC of thrombin time for predicting DC was 0.7803 (95%CI: 0.6411–0.9196), *P* = 0.0007 (Figure 2).

### 3.7. Efficacy Analysis of Blood Biochemical Indexes Combined with Coagulation-Related Indexes in Predicting DC

The cystatin C, blood chloride ion, fibrinogen, D-dimer, and thrombin time were selected, and ROC was used to analyze the efficacy of combined detection of cystatin C, blood chloride ion, fibrinogen, D-dimer, thrombin time in predicting the occurrence of DC. The results showed that the AUC of ROC was 0.9441 (95%CI: 0.8926–0.9957) (*P* < 0.001) (Figure 3).

## 4. Discussion

This retrospective study found that male gender and diabetes were independent risk factors for DC in the Chinese population. In addition, by analyzing the test results of blood biochemical indicators and the data of coagulation-related indicators, we found that cystatin C, blood chloride ion, fibrinogen, D-dimer, and thrombin time had relatively high predictive power for the occurrence of DC. At present, no studies have reported the correlation of blood biochemical indexes and coagulation-related indexes with DC. This research has opened up a precedent for this and has played an important role in the prevention and treatment of DC.

Current treatment options for DC include collagenase injection, acupuncture aponeurectomy, and fasciectomy. But complications and their incidence vary with each treatment option. Common complications include finger nerve/artery injury, flexor tendon injury, and wound healing complications such as hematoma, flushing reaction, complex local pain, and infection. [12]. Usually, DC patients should undergo surgery when there is an indication for surgery, which is easy to correct the deformity but still faces great difficulties in postoperative recurrence. Therefore, it is necessary to study the risk factors for the occurrence of DC and to find potential markers.

Diabetes appears to have long been recognized as a risk factor for the development of DC, although the exact mechanism has not been fully understood [11, 13]. The results of a meta-analysis found that the proportion of diabetes in DC patients was significantly higher than that in control [14]. In addition, studies have found that the incidence of DC in diabetic patients is 10 times that of nondiabetic people, and DC is also considered to be one of the complications of diabetes. When treating DC patients, surgeons are often concerned about the possibility of diabetes [15]. We know that the advanced glycation end products formed in the long-term high glucose environment are one of the pathogenesis of chronic complications of diabetes, and the advanced glycation end products are related to the occurrence of fibroproliferative diseases [16–18]. Researchers have found that higher levels of advanced glycation end products in the palmar fascia of DC patients may lead to collagen deposition and increased stiffness [11, 19]. In addition, studies have reported that myofibroblasts, which are responsible for contracting the fingers, are significantly increased in people with diabetes [20]. The above studies may be the underlying mechanism of diabetes and DC.

At present, gender may also be one of the key factors affecting the occurrence of DC. For example, Rydberg et al. [21] found a strong correlation between apolipoprotein levels and the occurrence of DC in patients of different genders. Another study found that androgens can act on the palmar fascia and the expression level of androgen receptors in patients with DC was significantly higher than that in normal palms, suggesting that androgen response status is associated with a higher incidence of DC in male patients [22]. This indicates that differences in hormone levels in different gender populations may be the underlying mechanism leading to the occurrence of DC, which further expands our knowledge of DC.

At the same time, we also analyzed the commonly used models for predicting the occurrence of DC. We found that the conventional blood biochemical indicators, including cystatin C and blood chloride ion levels, have certain predictive power for DC, and both of the AUCs exceeded 0.75. The AUC predicted by coagulation indexes including fibrinogen, D-dimer and thrombin time were all above 0.77. These results support our use of routine blood biochemical and coagulation-related index detection to predict the possibility of DC occurrence. Although using this single indicator to predict the occurrence of DC is very one-sided, we analyzed the power of the combined detection of these indicators and found that the AUC was as high as 0.9441, showing the excellent predictive power of the combined detection. The results suggest that we can predict the occurrence of DC in advance by combining cystatin C, blood chloride, fibrinogen, D-dimer, and thrombin time detection. Therefore, relevant intervention methods should be adopted to avoid the pain caused by surgery and other treatment methods after the occurrence and progression of DC.

Nonetheless, the study has some shortcomings. First, the incidence of DC is small in the Chinese population, so we just collected a small sample size. Our findings need to be validated in a larger sample. Additionally, we were unable to categorize studies based on disease severity in DC patients. In addition, we have not been able to analyze the genetic background of different populations. According to studies, genetic factors play an important role in the occurrence of DC [23–25].

## 5. Conclusion

In this retrospective study, we found that male gender and diabetes were independent risk factors for the development of DC. We can predict the risk of DC through the detection of blood biochemical indicators and coagulation-related indicators, especially the combined detection of cystatin C, blood chloride, fibrinogen, D-dimer, and thrombin time in predicting the occurrence of DC has a certain value.

## Figures and Tables

**Figure 1:** Receiver operating curves (ROC) of cystatin C and blood chloride levels in predicting DC. (a) ROC of cystatin C levels predicting DC. (b) ROC of blood chloride level predicting DC.

**Figure 2:** ROC of coagulation-related indicators for predicting DC. (a) ROC of fibrinogen levels predicting DC; (b) ROC of D-dimer levels predicting DC; and (c) ROC of thrombin time level predicting DC.

**Figure 3:** Receiver operating curves (ROC) of combined detection of cystatin C, blood chloride, fibrinogen, D-dimer, and thrombin time for predicting DC.

**Table 1:** Comparison of clinical data of DC patients and control group.

	DC (*n* = 21)	Control (*n* = 31)	Statistical value	*P* value
Age(year)			1.979	0.160
<60	6 (28.57%)	4 (12.90%)		
≥60	15 (71.43%)	27 (87.10%)		
Sex			17.164	<0.001
Male	17 (80.95%)	7 (22.58%)		
Female	4 (19.05%)	24 (77.42%)		
BMI (kg/m^2^)			1.456	0.228
<25	15 (71.43%)	17 (54.84%)		
≥25	6 (28.57%)	14 (45.16%)		
Smoking			4.510	0.034
No	14 (66.67%)	28 (90.32%)		
Yes	7 (33.33%)	3 (9.68%)		
Drinking			8.071	0.005
No	13 (61.90%)	29 (93.55%)		
Yes	8 (38.10%)	2 (6.45%)		
Hypertension			0.007	0.935
No	14 (66.67%)	21 (67.74%)		
Yes	7 (33.33%)	10 (32.26%)		
Diabetes			4.705	0.030
No	15 (71.43%)	29 (93.55%)		
Yes	6 (28.57%)	2 (6.45%)		
Coronary heart disease			2.157	0.142
No	21 (100%)	28 (90.32%)		
Yes	0 (0%)	3 (9.68%)		

DC: Dupuytren's contracture; BMI: body mass index.

**Table 2:** Analysis of risk factors for the occurrence of DC.

	*B*	SE	Wald	df	Sig.	Exp (*B*)	95%CI	
							Lower	Upper
Male gender	2.98	0.94	10.06	1	0.002	19.69	3.12	124.19
Age ≥60 years	−1.67	0.94	3.14	1	0.08	0.19	0.03	1.19
BMI ≥25 kg/m^2^	−1.09	0.75	2.09	1	0.15	0.34	0.08	1.47
Hypertension	−0.57	0.83	0.47	1	0.50	0.57	0.11	2.90
Diabetes	2.03	0.92	4.84	1	0.03	7.61	1.25	46.47
Smoking	0.33	1.02	0.10	1	0.75	1.39	0.19	10.16
Drinking	−1.53	1.02	2.25	1	0.13	0.22	0.03	1.60

DC: Dupuytren's contracture; CI: confidence interval.

**Table 3:** Comparison of blood biochemical index levels between DC patients and control groups (mean ± SD).

	DC (*n* = 21)	Control (*n* = 31)	*t* value	*P* value
Albumin (g/L)	42.21 ± 3.24	41.30 ± 2.80	1.079	0.286
Cystatin C (mg/L)	0.64 ± 0.09	0.58 ± 0.10	2.209	0.032
Creatinine (*μ*mol/L)	61.70 ± 10.82	56.28 ± 12.56	1.612	0.113
Alanine aminotransferase (U/L)	20.55 ± 15.48	18.09 ± 10.08	0.642	0.526
Aspartate aminotransferase (U/L)	24.05 ± 11.71	18.44 ± 6.54	1.995	0.056
Total bilirubin (*μ*mol/L)	13.68 ± 9.34	11.43 ± 4.23	1.034	0.310
Direct bilirubin (*μ*mol/L)	4.53 ± 2.76	4.27 ± 1.29	0.403	0.690
Indirect bilirubin (*μ*mol/L)	9.16 ± 7.06	7.17 ± 3.03	1.218	0.235
Total bile acids (*μ*mol/L)	7.87 ± 8.13	5.98 ± 5.81	0.979	0.332
Total cholesterol (mmol/L)	4.85 ± 1.19	4.78 ± 0.91	0.240	0.811
Triglycerides (mmol/L)	1.86 ± 1.93	1.38 ± 0.68	1.095	0.285
HDL-C (mmol/L)	1.41 ± 0.40	1.36 ± 0.28	0.531	0.598
LDL-C (mmol/L)	3.02 ± 0.94	3.04 ± 0.81	0.082	0.935
Glucose (mmol/L)	5.70 ± 1.00	5.58 ± 1.01	0.422	0.675
Blood urea nitrogen (mmol/L)	4.92 ± 1.28	5.24 ± 1.40	0.837	0.407
Creatinine (*μ*mol/L)	61.70 ± 10.82	56.28 ± 12.56	1.612	0.113
Uric acid (*μ*mol/L)	289.30 ± 73.50	269.09 ± 76.03	0.953	0.345
Potassium (mmol/L)	4.13 ± 0.49	3.89 ± 0.31	1.991	0.055
Sodium (mmol/L)	140.84 ± 2.39	140.88 ± 1.26	0.070	0.944
Chlorine (mmol/L)	102.00 ± 2.89	104.78 ± 1.98	4.122	<0.001

DC: Dupuytren's contracture; HDL-C: high-density lipoprotein cholesterol; LDL-C: low-density lipoprotein cholesterol.

**Table 4:** Comparison of coagulation-related indexes between DC patients and control groups (mean ± SD).

	DC (*n* = 21)	Control (*n* = 31)	*t* value	*P* value
Fibrinogen	2.83 ± 0.53	3.59 ± 0.86	3.939	<0.001
D-dimer	0.29 ± 0.14	1.10 ± 1.04	4.280	<0.001
Thrombin time	14.26 ± 2.23	12.63 ± 1.28	3.029	0.005

DC: Dupuytren's contracture.

## Data Availability

Clinical data for this study can be obtained from the corresponding author upon request.
